# Prediction of Conversion from CIS to Clinically Definite Multiple Sclerosis Using Convolutional Neural Networks

**DOI:** 10.1155/2022/5154896

**Published:** 2022-07-15

**Authors:** H. M. Rehan Afzal, Suhuai Luo, Saadallah Ramadan, Manju Khari, Gopal Chaudhary, Jeannette Lechner-Scott

**Affiliations:** ^1^School of Electrical Engineering and Computing, University of Newcastle, Callaghan, NSW 2308, Australia; ^2^Hunter Medical Research Institute, New Lambton Heights, NSW 2305, Australia; ^3^Jawaharlal Nehru University, New Delhi, India; ^4^Bharati Vidyapeeth College of Engineering, New Delhi, India; ^5^Department of Neurology, John Hunter Hospital, New Lambton Heights, NSW 2305, Australia

## Abstract

Multiple sclerosis (MS) is a chronic neurological disease of the central nervous system (CNS). Early diagnosis of MS is highly desirable as treatments are more effective in preventing MS-related disability when given in the early stages of the disease. The main aim of this research is to predict the occurrence of a second MS-related clinical event, which indicates the conversion of clinically isolated syndrome (CIS) to clinically definite MS (CDMS). In this study, we apply a branch of artificial intelligence known as deep learning and develop a fully automated algorithm primed with convolutional neural network (CNN) that has the ability to learn from MRI scan features. The basic architecture of our algorithm is that of the VGG16 CNN model, but amended such that it can handle MRI DICOM images. A dataset comprised of scans acquired using two different scanners was used for the purposes of verification of the algorithm. A group of 49 patients had volumetric MRI scans taken at onset of the disease and then again one year later using one of the two scanners. In total, this yielded 7360 images which were then used for training, validation, and testing of the algorithm. Initially, these raw images were taken through 4 steps of preprocessing. In order to boost the efficiency of the process, we pretrained our algorithm using the publicly available ADNI dataset used to classify Alzheimer's disease. Finally, we used our preprocessed dataset to train and test the algorithm. Clinical evaluation conducted a year after the first time point revealed that 26 of the 49 patients had converted to CDMS, while the remaining 23 had not. Results of testing showed that our algorithm was able to predict the clinical results with an accuracy of 88.8% and with an area under the curve (AUC) of 91%. A highly accurate algorithm was developed using CNN approach to reliably predict conversion of patients with CIS to CDMS using MRI data from two different scanners.

## 1. Introduction

MS is a chronic inflammatory disease of the central nervous system (CNS) [1]. It is considered to be an autoimmune disease, with lymphocytes attacking the CNS resulting in demyelination, inflammation, and axonal damage. Damage to the CNS can involve simultaneously several different areas. The World Health Organization (WHO) reports that currently there are more than 2 million MS sufferers globally, with the disease having an estimated prevalence of 30 cases per 100,000 people worldwide. The average age of sufferers is 29.2 years, and the rate of disease in people between the ages 25.3 and 31.8 is increasing rapidly. MS seems to occur more frequently in women, and the ratio seems to be increasing steadily [2].

There is no specific diagnostic method for MS, with diagnoses usually being made based on an assessment of a patient's symptoms, MRI scans of white matter lesions, and the exclusion of other diseases. Generally, patients initially present with clinically isolated syndrome (CIS), in which MS-like symptoms are apparent, but a definite diagnosis cannot always be made. For around 20% of CIS patients, the initial event is isolated and remains so, with no further progression even after two decades [3]. However, around 30% of CIS patients will get a second attack and (thus) a diagnosis of CDMS within one year. Certain criteria have been developed to assist in the diagnosis of MS, the most recent being McDonald et al.'s criteria [4]. Barkhof et al.'s [5] and MAGNIMS guidelines [6] help in determining MS characteristics on MRI. These guidelines were developed to be able to include patients early into clinical trials but are not always helpful in clinical practice.

Apart from its application in the diagnosis of MS, MRI is used also to follow a patient's progress. In this regard, specific MRI sequences based on different tissue contrasts are used in order to highlight particular tissue changes. For example, fluid-attenuated inversion recovery (FLAIR) images achieve the best visualization of MS plaques, while *T*1 weighted (*T*1w) is considered the most reliable when measurements of atrophy are required [7].

Interest in a subset of AI known as deep learning has been increasing in medicine in recent years due to the predictive accuracy and robustness that it offers. Deep learning has a range of medical applications, with one of these being in the segmentation of MRI scans [8–15]. While artificial intelligence and specifically its subbranches of machine learning and deep learning are being used in the classification and prognosis of MS, the work done in this area remains limited. So, we have tried to overcome this issue by developing a fully automated algorithm.

In this study, we have attempted to overcome the problems relating to robustness and accuracy described above with a fully automated method that uses VGG16 with CNN architecture that we have especially modified. We developed an earlier algorithm for the prediction of CIS to CDMS [16]. These preliminary results were derived from a small dataset and had a simple architecture. The algorithm predicted the presence of MS with an accuracy of 83.3% and 100% in two experiments with different settings. We improved this earlier algorithm by using a bigger dataset and developed a new automated complex algorithm trained especially for DICOM images. This new algorithm is now tested on more scans and has robust and reliable architecture as described in the next section. Convolutional neural networks (CNNs) were applied to predict the conversion of CIS patients to CDMS within the first year.

## 2. Methodology

We modified the architecture of our preexisting VGG16 algorithm to enable it to handle 3D volumetric MRI scans in the DICOM format. This modified algorithm was then pretrained on an ADNI [17] dataset in order to obtain initial weights. Two separate datasets consisting of conventional MRIs acquired from a group of MS patients using two different scanners were preprocessed before then being used to train the algorithm. These datasets will be described in detail in the following sections. The method described above not only allowed us to achieve a high level of accuracy but was also very robust in nature due to the approach of using datasets acquired from two different scanners. This automated algorithm will help neurologists to diagnose MS at an early stage when treatment is most efficacious. A general diagram of the algorithm can be seen in Figure 1.

### 2.1. Dataset

Evaluation of the algorithm was done using datasets from two different MRI scanners. One of these datasets consisted of scans from 21 patients at each of two time points (CIS and a 1-year follow-up—42 scans in total) at the Hunter Medical Research Institute Imaging Centre (HMRI-IC) using a Siemens PRISMA 3T MRI scanner. Clinical evaluation after one year using McDonald et al.'s criteria indicated that 11 of these patients had converted to CDMS, and 10 had not. The other dataset consisted of scans acquired from 28 patients at each of two time points (CIS and a 1-year follow-up—56 scans in total) at the John Hunter Hospital (JHH) using a Siemens 3T VARIO MRI scanner. Clinical evaluation after one year using McDonald et al.'s criteria indicated that 15 of these patients had converted to CDMS and 13 had not by that time. Both *T*1w and FLAIR scanning sequences were used in the acquisition of each of the datasets above. Importantly, the use of two different scanners for the acquisition of data allowed us to test the robustness of our method.

From the above, 3D scans taken from 49 CIS patients at one time point and then again at a second time point one year later gave a total of 98 MRI volumetric scans, which at an average of 80 slices per MRI scan yielded 7360 images. Clinical evaluation of patients at the second time point revealed that 26 had converted to CDMS and 23 had not. The scans of 40 of these patients were then used to train the algorithm, with this training dataset then being randomly divided into subsets for training and validation at a ratio of 80 : 20. Scans from the remaining 9 patients were used for testing purposes. These datasets are presented in more detail in Table 1.  Figure 2 gives the percentage relative sizes of the training, validation, and testing datasets.

### 2.2. Preprocessing

The two datasets were preprocessed using statistical parametric mapping (SPM) [18]. Preprocessing helps us to improve the results by denoising and normalization of the images. Preprocessing steps included skull stripping, intensity normalization, image denoising, and image registration. For skull stripping, we used a Brain Extraction Tool (BET) by Salehi et al. [19]; for intensity normalization, we used N3 intensity normalization by Leger et al. [20]; while for image denoising, we used Gaussian presmoothing filters. Rigid registration was performed using a Functional Magnetic Resonance Imaging of the Brain (FMRIB) Linear Image Registration Tool (FLIRT).

### 2.3. Pretraining and Data Augmentation

Before the MS datasets were uploaded to the algorithm, we implemented two important steps: an algorithm pretraining step and a data augmentation step. These techniques were applied in order to compensate for size limitations in our MS datasets.

It can be difficult for naïve CNN models to learn the general relevance of features, so because the limited size of our MS datasets precluded us from using them to train our algorithm from scratch, we undertook pretraining of the algorithm using 921 scans from the publicly available ADNI datasets. These 921 scans were made up of 276 scans from either normal subjects or Alzheimer's patients and were taken at multiple sites at from 1 to 3 time points using a variety of 1.5 Tesla scanners. Pretraining of our algorithm using this data gave us initial weights, which could then be used for the main training of the algorithm using our MS training dataset. This pretraining is a type of transfer learning which can lead to improvements in classification results when only limited data is available. Transfer learning is a technique in which a model that has already been developed for a particular task is used as the starting point for the development of another model needed for a different task.

Data augmentation is used to increase the amount of data in a limited dataset through the addition of modified copies of existing data or synthetic data to the dataset. Bigger datasets allow better training of algorithms and also reduce the risk of overfitting in complex algorithms such as our amended algorithm. We applied data augmentation techniques including cropping, flipping, translating, scaling, and rotating to both the PRISMA and VARIO datasets. Preprocessing steps such as intensity inhomogeneity, gradient nonlinearity, and phantom-based distortion correction had already been done on these scans before data augmentation was applied.

### 2.4. CNN Architecture

VGG16's architecture [21] comprises thirteen convolutional layers, three fully connected (FC) layers, and a softmax layer for prediction purposes. It was designed by the Visual Geometry Group (VGG) of London, mainly for the purposes of classification. One reason why this is a popular algorithm is that it comes with weights provided. These weights allow researchers to fine tune the algorithm based on its intended application, which in our case is medical imaging.

A 3 × 3 kernel is used as a sliding window which is passed over the images at each of the 13 convolutional layers. The stride value controls the degree of slide, which could, for example, be pixel by pixel or could skip a certain number of pixels as per requirements. The general equation for learning features as the window slides over an image can be expressed as follows:

(1) $$\begin{array}{c} y=f\left(Lx+B\right), \end{array}$$

where *L* and *B* are the learnable parameters, *x* is the pixel value, and *y* is the output.

Each of the 13 convolutional layers has a range of 3 × 3 filters and is associated with an activation layer—that being a rectified linear unit (ReLU) in our case. MaxPooling was used for the downsampling of the features. These layers are used for the automatic extraction of features, which in our case are features that will allow us to discriminate between patients who will go on to develop MS and those who will not. This extraction of features yields features maps, and some examples of which are shown in Figure 3. After the convolutional layers comes the fully connected (FC) layer, which is the penultimate layer and acts as a classifier. Finally, we have the softmax function which calculates the probability that the images are from a patient who will go on to develop MS.

VGG was made with a greater number of layers and smaller filter sizes than other classification algorithms specifically so that it could be used in the learning of more complex features, and all this leads to a generally more complex system. Appropriate management can ensure that this system can yield better results than less complex architectures. We used data augmentation to increase the quantity and variety of our images, which yielded output with better accuracy. All images were resized to 224 × 224 before being input into the algorithm so as to maintain consistency of input across both datasets.

After testing a variety of different window configurations and stride values, we settled on a 3 × 3 sliding window with a stride value of 1. The smaller window size was chosen, and we found that larger windows result in more false positives.

With the above modifications to our algorithm, we were able to identify a greater variety of features at an increased resolution than would be possible using the VGG model. MS lesions can be very small and typically occupy only around 1% of the total brain volume, so the more sensitive the method for their detection, the better. Currently, neurologists mostly depend on the visual application of McDonald et al.'s criteria to MRI scans when trying to identify the types of brain lesion that will allow them to differentiate between MS and non-MS patients. Our algorithm will allow the automatic selection of dense features and will so assist in the efficient classification of scans as either diseased or nondiseased.

## 3. Implementation Details

Our algorithm was written in Python, using Keras with TensorFlow at the back-end due to their open-source nature and associated range of machine learning libraries. We used a 2.7 GHz Intel Xeon Gold processor (model no. E5-6150) with a 32 GB Nvidia GPU. The method was run for 120 epochs, with early stopping for a patience value of 15. We set the batch size at 64, and the learning rate at 0.0001. The algorithm was run using Da's method [22] as an optimizer.

### 3.1. Evaluation Metrics

A range of metrics was used to check the accuracy of our method. These metrics were used on both datasets and are defined as follows.

#### 3.1.1. Accuracy

The accuracy of the algorithm is calculated by the following formula:

(2) $$\begin{array}{c} \text{Accuracy}=\frac{T_{P}+T_{n}}{p+n}, \end{array}$$

where *T*_*p*_represents the number of true positives, *T*_*n*_ represents the number of true negatives, and (*p* + *n*) is the total population.

#### 3.1.2. Precision

Precision (also known as the lesion false discovery rate—LFPR) is defined by the following:

(3) $$\begin{array}{c} \text{Precision}=\frac{T_{p}}{T_{p}+F_{p}}, \end{array}$$

where *F*_*p*_ represents the number of false positives.

#### 3.1.3. Recall/Sensitivity

The recall/sensitivity of the method (also known as the lesion true positive rate—LTPR) is defined by the following:

(4) $$\begin{array}{c} \frac{\text{Recall}}{\text{Sensitivity}}=\frac{T_{p}}{T_{p}+F_{n}}, \end{array}$$

where *F*_*n*_ is the number of false negatives.

#### 3.1.4. DSC/*F*1 Score

The overall accuracy of the algorithm as expressed in terms of the dice similarity coefficient (DSC) between automated segmentation masks and manually annotated areas is defined by the following:

(5) $$\begin{array}{c} \frac{\text{DSC}}{F1}\text{score}=\frac{2\times T}{F_{n}+F_{p}+2\times T_{p}}. \end{array}$$

### 3.2. Results

Training of our algorithm resulted in the identification of a range of features, and some examples of which are shown in Figure 3.  Figure 4 shows some heat maps of scans classified by our algorithm. Heat maps such as these are used to show the positive and negative relevance of the algorithm's results. The green areas correspond to lesions that have been correctly classified by the algorithm, while the red areas correspond to incorrectly classified (i.e., false positive) areas. We were able to achieve training and validation accuracies for our algorithm of 85% and 83%, respectively. The manual segmentation was used as gold standards. The accuracy graph is shown in Figure 5, and the area under the curve (AUC) is shown in Figure 6. The AUC was calculated as 91%. As previously mentioned, scans from 9 of the patients were used for testing purposes. A range of metrics was applied to each of these scans, and the averages were calculated (see Table 2). All evaluation metrics are shown in Figure 7.

## 4. Discussion

The robustness of our algorithm is shown in its ability to maintain high accuracy for prediction of disease throughout both the PRISMA and VARIO datasets. Further evidence for this robustness lies in the stability of the accuracy, *F*1 score, precision, and recall parameters for data taken at different time points and with different scanners.

Our qualitative and quantitative results are improved compared to previously published algorithms. Wottschel et al. [23] developed an algorithm that used machine learning techniques to predict the conversion of CIS to CDMS. Their dataset consisted of seventy-four patients at CIS stage, with the scans being clinically reviewed after one year and three years. Scans of confirmed CDMS patients were used as their benchmark with a support vector machine (SVM) being used with the purpose of classification and prediction. They implemented a multimodel architecture in which the patient's demographic and clinical data were used together with conventional MRI. Clinical evaluation showed that 30% of the patients had converted to MS after one year, and 44% had converted after three years. The SVM's accuracy in predicting patient conversion to CDMS after one year was only 71.4% with a sensitivity of 77% and a specificity of 66%, while the accuracy for predicting patient conversion after 3 years was worse at only 60% with a specificity of 76%. This algorithm had limitations, as accuracy was very low, and after three years, it was even worse.

Another algorithm with the same aim was described by Zhang et al. [24], and they developed an algorithm based solely on an imaging-based machine learning technique (i.e., random forest) to predict the conversion of CIS to CDMS. The success of their algorithm was limited due to their lack of a multimodel approach. Their dataset consisted of scans acquired from a single cohort of 84 patients from one site, with a follow-up at three years. McDonald et al.'s criteria were used for the clinical classification of MS patients. After completing computer-assisted manual annotation of lesions, they used SPM for automatic segmentation of lesions and then identified the brightness features and the shape features from the segmented masks. These features were then used as input for their algorithm when training the random forest classifier, which was then able to predict conversion to MS with an accuracy of 84.5%. Their research suggested that shape features were useful in predicting MS, whereas intensity features were of little help. Like the previously discussed algorithm, this algorithm also has its limitations. The limitation of their approach was that the accuracy of their algorithm was checked by using only one type of scanner at only one site (the same scanner in fact), which meant that the robustness of their algorithm was not tested.

Eitel et al. [25] proposed an algorithm using CNN to diagnose MS by using conventional MRI and a layer-wise propagation technique for CNNs. The architecture was pretrained like in our study on the publicly available Alzheimer's Disease Neuroimaging Initiative (ADNI) dataset, which consists of 921 scans of Alzheimer patients. Their study involved a cohort of 147 subjects, which included both MS patients and healthy controls, with CNN being used to distinguish between the two groups. They were able to achieve an accuracy of 87.04% to differentiate MS from healthy controls using their architecture, concluding that their CNN model was able to diagnose MS with considerable accuracy but did not determine the prediction of conversion from CIS to MS. Also, as with the study previously mentioned, the robustness of their algorithm remained untested.

In our developed algorithm, we focused on robustness by including datasets from different scanners. Two different scanners had different parameters which were handled by preprocessing. Image registration was performed to align all images, and then, training was performed. In this study, we developed a fully automated algorithm primed with convolutional neural network (CNN) that has the ability to learn the features of MRI scans. The basic architecture of our algorithm is that of the VGG16 CNN model, but amended such that it can handle MRI DICOM images. A dataset comprised of scans acquired using two different scanners was used for the purposes of verification of the algorithm. The qualitative and quantitative results above indicate that our fully automated algorithm is able to predict conversion to MS with an accuracy of 88.8% robust in nature as it was checked on different scanners and different deep learning parameters, which suggests that it could have a role as a valuable time saving tool for neurologists.

The main limitation of our study is the limited dataset as deep learning works best with extremely large datasets. In future, we will collect more datasets from different scanners that will help us to increase the efficiency of our algorithm. We also plan to train our algorithm on multimodal data, including demographic and clinical data. This algorithm will also be checked with different parameters like different batch sizes, different convolutional layers, filters, and learning rate according to that dataset. More sequences of MRI will be added to increase accuracy and reliability of algorithm.

## 5. Conclusion

In this study, we describe a fully automated algorithm for the early diagnosis of MS. This algorithm predicts whether a CIS patient will go on to develop CDMS within one year. Our method involved three main steps. The first of these is a 4-step preprocessing of a MS dataset by SPM. This is followed by pretraining of the algorithm using the publicly available ADNI dataset and then training of the algorithm using the preprocessed MS dataset. This approach, which is an example of transfer learning, can improve the quality of results if only a limited dataset is available. In our case, this was facilitated through the use of data augmentation to generate more scans from our limited datasets. Our results have shown that our amended VGG16 algorithm works very well for medical imaging. Accuracy of the algorithm was tested by applying a range of valuation metrics including accuracy, *F*1 score, recall, and precision across the two MS datasets. The efficacy of the algorithm was borne out by quantitative as well as qualitative results, which we have presented along with relevant graphs in Results. This automated algorithm will help neurologists to predict whether or not CIS patients will progress to CDMS within the first year and so allow early interventions.

## Figures and Tables

**Figure 1:** General diagram of the algorithm developed in this study.

**Figure 2:** Percentage of scans (combined PRISMA/VARIO dataset) used for training, validation, and testing.

**Figure 3:** Some examples of feature maps.

**Figure 4:** Examples of heat maps, where the green color shows the true positives and the red color shows the false positives.

**Figure 5:** Accuracy graph for the algorithm.

**Figure 6:** AUC curve for the algorithm (AUC = 91%).

**Figure 7:** Evaluation metrics for the algorithm.

**Table 1:** PRISMA and VARIO datasets.

	PRISMA	VARIO
Training	17	23
Testing	4	5
Total	21 (42)	28 (56)
Types	*T*1w, FLAIR	*T*1w, FLAIR

42 and 56 show two time points, one is at CIS and one is at CDMS, and make 98 MRI scans in total, where every MRI has 80 average slices which make 7360 images in total.

**Table 2:** Different evaluation metrics for training, validation, and testing.

Process	Accuracy (%)	Recall (%)	Precision (%)	*F*1 score (%)
Training	89.0	—	—	—
Validation	83.0	—	—	—
Testing	88.8	76.0	86.3%	79.5

## Data Availability

Dataset is publicly not available due to Australian government regulations because data used in training and testing of algorithms is collected from local hospitals in Australia.
